The article "Long non-coding RNA ZFY-AS1 represses periodontitis tissue inflammation and oxidative damage via modulating microRNA-129-5p/DEAD-Box helicase 3 X-linked axis" was retracted in 2026. Reasons: concerns about the data; concerns about the results or conclusions.

# Long non-coding RNA ZFY-AS1 represses periodontitis tissue inflammation and oxidative damage via modulating microRNA-129-5p/DEAD-Box helicase 3 X-linked axis

**DOI:** 10.1080/21655979.2021.2019876

**Published:** 2022-06-05

**Authors:** Lin Cheng, YuLing Fan, Jue Cheng, Jun Wang, Qingmei Liu, ZhiYuan Feng

**Affiliations:** a Department of Stomatology, Bethune Hospital, (Shanxi Academy of Medical Sciences), Taiyuan City, Shanxi Province, China; b Department of Stomatology, School of Stomatology, Shanxi Medical University, Taiyuan City, Shanxi Province, China; c Department of Stomatology, The Community Health Service Center of Beijing Jiao Tong University, Beijing City, China; d Department of Orthodontics, Shanxi Provincial People’s Hospital, Taiyuan City, Shanxi Province, China

**Keywords:** Long non-coding RNA ZFY-AS1, microRNA-129-5p, periodontitis, oxidative damage

## Abstract

A large number of studies have manifested long non-coding RNA (lncRNA) is involved in the modulation of the development of periodontitis, but the specific mechanism has not been fully elucidated. The purpose of this study was to explore the biological function and latent molecular mechanism of lncZFY-AS1 in periodontitis. The results clarified lncZFY-AS1 and DEAD-Box Helicase 3 X-Linked (DDX3X) were up-regulated, but microRNA (miR)-129-5p was down-regulated in periodontitis. Knockdown of lncZFY-AS2 or overexpression of miR-129-5p decreased macrophage infiltration and periodontal membrane cell apoptosis, increased cell viability, repressed inflammatory factors and nuclear factor kappa B activation, reduced oxidative stress, but promoted nuclear factor-E2-related factor 2/heme oxygenase 1 expression. LncZFY-AS1 elevation further aggravated periodontitis inflammation, oxidative stress, and apoptosis. LncZFY competitively adsorbed miR-129-5p to mediate DDX3X expression. Knockdown lncZFY’s improvement effect on periodontitis was reversed by depressive miR-129-5p or enhancive DDX3X. In conclusion, these data suggest lncZFY-AS1 promotes inflammatory injury and oxidative stress in periodontitis by competitively binding to miR-129-5p and mediating DDX3X expression. LncZFY-AS1/miR-129-5p/DDX3X may serve as a novel molecular target for treatment of periodontitis in the future.

## Highlights

- LncZFY-AS1 and DDX3X were upregulated in periodontitis, while miR-129-5p was down-regulated;
- Repressive lncZFY-AS2 or elevated miR-129-5p reduced LPS-induced periodontal membrane cell inflammation, oxidative damage, and inflammation;
- Overexpressed lncZFY-AS1 or knockdown miR-129-5p aggravated periodontitis inflammation, and oxidative stress and apoptosis;
- The improvement of depressive lncZFY on periodontitis was reversed via knockdown miR- 129-5p or elevated DDX3X;
- LncZFY competitively absorbed miR-129-5p to mediate DDX3X expression.

The article "Long non-coding RNA ZFY-AS1 represses periodontitis tissue inflammation and oxidative damage via modulating microRNA-129-5p/DEAD-Box helicase 3 X-linked axis" was retracted in 2026. Reasons: concerns about the data; concerns about the results or conclusions.

## 1. Introduction

Periodontitis is a long-term inflammatory illness featured via swollen gums, reduced absorption of alveolar bone and loosening of teeth. It has become the major reason of tooth loss in adults [1]. Periodontitis is mainly induced via microbial infections like *porphyromonas gingivalis* (*Pg*) [2]. Microbial infection is available to induce severe inflammation, and result in gum tissue damage, thus leading to abscission. Meanwhile, numerous studies have clarified that microbial infection is available to expedite the production of reactive oxygen in the periodontal part and destruct the balance of oxidation with antioxidant, thus further aggravating gingival damage [3]. At present, the cure approaches of periodontitis mainly consist of antibiotic treatment, the dental cleaning and surgery, but the therapeutic impacts still require to be perfected [2,4]. Hence, it is crucial to further understand the pathogenesis of periodontitis and seek brand-new molecular therapeutic targets.

Long non-coding RNAs (lncRNAs) are a group of RNAs not encoding proteins. But recently, it has been discovered that they are available to prevent microRNAs (miRNAs) from combining with proteins via absorbing miRNAs, thus functioning in post-transcriptional modulation [5,6]. Elevated studies have reported aberrant lncRNAs in periodontitis and the participation of them in the process of modulating periodontitis progression. For instance, Li J *et al*. discover that lncRNA Nron effectively restrains osteoclast formation and alveolar bone resorption in periodontitis and accelerates nuclear transport of nuclear factor kappa B (NF-κB) inhibitor [7]. Recently, a high-throughput sequencing study manifests that a brand-new lncRNA, lncZFY-AS1 is enhancing in periodontitis [8]. However, the biological function and molecular mechanism of lncZFY-AS1 in periodontitis remain ambiguous.

A large number of studies have manifested lncRNA and target protein compete for the binding site of miRNA, so as to exert the post-transcriptional regulation of modulatory protein-coding genes [9]. For example, lncDCST1-AS1 curbs the proliferation of periodontal membrane cells (PDLCs) via adsorption of miR-21 and augment of periodontal ligament-associated protein-1 (PLAP-1) [10]. A study also elucidates lnc01126 expedites inflammation and apoptosis of PDLCs cells via modulating miR-518a-5p/hypoxia inducible factor-1α (HIF-1α)/mitogen-activated protein kinase (MAPK) pathway [11].

MiRNAs are also members of non-coding RNAs and are manifested in large quantities in biological tissues or cells [12]. Former studies have clarified that miRNA is momentous in the modulation of periodontitis inflammation [13], oxidative stress [14], autophagy and bone resorption [15]. It refrains the biological function of target proteins majorly via combining with downstream target genes [12,16]. MiR-129-5p is a part of the miRNA family. A recent study has discovered that miR-129-5p refrains nonalcoholic fatty liver inflammation and fibrosis via combining with downstream Suppressor of cytokine signaling 2 (SOCS2) proteins [17]. Huang X *et al*. discover that miR-129-5p mitigates lipopolysaccharide (LPS)-induced acute kidney injury via controlling downstream Toll-like receptors and NF-κB pathway [18]. Meanwhile, miR-129-5p lightens oxidative stress and inflammation in heart failure via combining with high mobility group box-1 (HMGB1) protein. However, the biological function of miR-129-5p in periodontitis remains uncertain.

The article "Long non-coding RNA ZFY-AS1 represses periodontitis tissue inflammation and oxidative damage via modulating microRNA-129-5p/DEAD-Box helicase 3 X-linked axis" was retracted in 2026. Reasons: concerns about the data; concerns about the results or conclusions.

In this study, examination of lncZFY-AS1 and miR-129-5p was in periodontitis mice and cell models, and exploration of the impacts of knockdown or enhancive lncZFY-AS1 and miR-129-5p on periodontitis inflammation and oxidative stress was conducted. Meanwhile, in this study, further exploration of the latent molecular mechanism of lncZFY-AS1/miR-129-5p was in modulating periodontitis injury. This study may offer brand-new strategies and targets for periodontitis cure.

## 2. Materials and methods

### 2.1 Clinical sample collection

From May 2017 to November 2019, gain of gingival tissues of 54 periodontitis patients and 23 healthy controls was from Bethune Hospital, (Shanxi Academy of Medical Sciences). Collection of gingival tissue samples was from patients with periodontitis within gingivectomy during orthodontic or prosthodontic treatment and from healthy subjects during crown lengthening. Approval of this study was via the Ethics Committee of Bethune Hospital, (Shanxi Academy of Medical Sciences) and gain of written informed consent was from the subjects.

### 2.2 Mouse model of periodontitis

Establishment of the mouse periodontitis model was as set forth [19]. Performance of oral infection was via *Pg* bacterial strain (ATCC: 33277) and growth of the bacteria was in an anaerobic chamber at 37°C (80% N_2_, 10% H_2_, and 10% CO_2_). Addition of Kanamycin (0.5 mg/mL) was to drinking water for 3 consecutive days to remove other bacteria prior to formal oral bacterial colonization. Mixing of bacterial precipitate gained via centrifugation was with equal volume of sterile 3% carboxymethyl cellulose and topical application to the mouth and anus was for eight consecutive times. The dosage of the mixture was 100 μL (5 × 10^10^ cells/mL of *Pg*) per mouse. After bacterial application, chicken type II collagen (Cat#20011, Chondrex) was emulsified in 100 μg complete freund’s adjuvant (Cat#7023, Chondrex). A slow intradermal injection of 50 µL emulsion was made at a point about 1.5 cm away from the root of the tail. Primary immunization was conducted 1 day after vaccination and booster immunization was performed 14 d later.

The article "Long non-coding RNA ZFY-AS1 represses periodontitis tissue inflammation and oxidative damage via modulating microRNA-129-5p/DEAD-Box helicase 3 X-linked axis" was retracted in 2026. Reasons: concerns about the data; concerns about the results or conclusions.

### 2.3 Grouping of animals

Raising of the mice was in standard laboratory animal facilities with giving basic food and water. All animal experiments obeyed the Guidelines for Animal Research: Reporting of *In Vivo* Experiments and the approval was via the Animal Care Committee of Bethune Hospital, (Shanxi Academy of Medical Sciences). Two days before *Pg* infection, injection of 200 μL sh-negative control (NC)/lncZFY-AS1 lentiviral plasmid vector (2 × 10^8^ TU/mL, GenePharma, Shanghai, China) was into the mice via the tail vein. Casual assignation of 28 mice was into four groups: the control (no ligation), the model (the mice received with *Pg* oral infection), the periodontitis + sh-lncZFY-AS1/NC (the mice received with *Pg* oral infection and injected with sh-lncZFY-AS1/NC lentivirus plasmids). Euthanasia of the mice was via inhaling excess CO_2_, and collection of periodontal tissue samples was done. Purchase of all BALB/c mice (male, 5–6 weeks old) was from Hunan SJA Laboratory Animal Co., Ltd. (Changsha, China).

### 2.4 Immunohistochemistry

Immunohistochemical staining was performed as set forth. For immunohistochemical staining, the tissues were fixed with 4% paraformaldehyde and decalcified in 10% ethylenediaminetetraacetic acid buffer. All samples were embedded in paraffin blocks and 4 μm sections were prepared. The sections were dewaxed and rehydrated. The sections were incubated with anti-LC3 antibody (1: 200; Abcam) and biotinylated goat immunoglobulin G (IgG). Finally, visualization of immune reactivity was conducted via diaminobenzidine (Beyotime, Shanghai, China).

### 2.5 Terminal deoxynucleotidyl transferase-mediated dUTP-biotin nick end labeling (TUNEL)

In order to intuitively observe the apoptosis of periodontal tissues, apoptotic cells were detected by TUNEL staining as mentioned above [20]. Processing of the sections and staining with TUNEL reactive mixture were in line with manufacturer’s instructions (Wanleibio Co., Ltd.). Staining of the cell nuclei was with 4ʹ, 6-diamidino-2-phenylindole solution. Observation of the sections was under a fluorescence microscope, and addition of anti-fluorescence quenching agent (Wanlei Biological Co., Ltd.) was conducted. Within 24 h, images of the sections were captured under a fluorescence microscope. Count of the apoptotic cells was via ImageJ Pro Plus 6.0 (NIH) and analysis of the results was manifested.

The article "Long non-coding RNA ZFY-AS1 represses periodontitis tissue inflammation and oxidative damage via modulating microRNA-129-5p/DEAD-Box helicase 3 X-linked axis" was retracted in 2026. Reasons: concerns about the data; concerns about the results or conclusions.

### 2.6 Cell culture

Gain of human periodontal membrane cells (hPDLCs) was performed as set forth [21]. The periodontal membrane was gently scraped from the root surface of healthy subjects and detached with collagenase and trypsin (Gibco, Grand Island, NY, USA). Culture of the cells was in Dulbecco’s Modification of Eagle’s Medium (Gibco, Carlsbad, CA, USA) with 10% fetal bovine serum (Gibco), 100 U/mL penicillin and 100 μg/mL streptomycin and in an incubator. Application of the 3^rd^ passage of hPDLCs was for subsequent experiments. For establishment of a model of periodontitis, treatment of PDLCs was with 100 ng/mL LPS (Sigma, St. Louis, MI, USA).

### 2.7 Cell transfection

Conduction of cell transfection was as formerly described [22]. Design and offering of small interfering RNAs targeting lncZFY-AS1 and DDX3X, NCs (si-NC/si-lncZFY-AS1/si-DDX3X) and elevated plasmids (pcDNA 3.1/pcDNA 3.1-lncZFY-AS1/pcDNA 3.1-DDX3X) were via GenePharma (Shanghai, China). Purchase of miR-129-5p mimic/inhibitor and its NC was from Integrated Biotech Solutions Co. (Shanghai, China). Seeding of hPDLCs was into 6-well plates, and after 80% confluence, transitive transfection of the plasmids or oligonucleotides was into hPDLCs via Lipofectamine 3000 (Invitrogen, Carlsbad, CA, USA) in line with the manufacturer’s protocol. After 48 h, harvest of the cells was for subsequent experiments.

### 2.8 Detection of oxidation and inflammatory indexes

Detection of malondialdehyde (MDA), superoxide dismutase (SOD), Catalase (CAT), Tumor necrosis factor-α (TNF-α), Interleukin (IL)-1β and IL-6 was in cells and tissues in line with kit method [23]. Purchase of the above kits was from Nanjing JianCheng Bioengineering Institute (Nanjing, China).

### 2.9 Cell viability

Measurement of cell viability was via 3-(4, 5-dimethylthiazol-2-yl)-2, 5-diphenyltetrazolium bromide (MTT) assay as described earlier [24]. Seeding of LPS-treated or transfected cells was into 96-well plates (1 × 10^4^ cells/well), and incubation of 5 μL MTT solution was to each well. Mixing Dimethyl sulfoxide solution (Sigma-Aldrich) with cells in each well, was to melt the reaction product formazan. Via a microplate reader (Molecular Devices; Hercules, CA, USA) was measured the absorbance at 570 nm.

### 2.10 Flow cytometry

In line with the manufacturer’s instructions, application of Annexin V- fluorescein isothiocyanate Apoptosis Detection Kit (YEASEN, Shanghai, China) was conducted. Collecting cells was for apoptosis detection. Resuspension of the cells was in binding buffer at a concentration of 1 × 10^6^ cells/mL. Addition of 5 μL Annexin-V and 10 μL propidium iodide was to every 100 μL of the resuspended cell solution, then incubation was manifested, and analysis was with a flow cytometer (Beckman Coulter, CA, USA).

The article "Long non-coding RNA ZFY-AS1 represses periodontitis tissue inflammation and oxidative damage via modulating microRNA-129-5p/DEAD-Box helicase 3 X-linked axis" was retracted in 2026. Reasons: concerns about the data; concerns about the results or conclusions.

### 2.11 Real-time fluorescent quantitative PCR (RT-qPCR)

Performance of RT-qPCR was as set forth [25]. TRIzol reagent (Invitrogen, USA) was applied to extract total RNA from cells and tissues in line with manufacturer’s instructions. A complementary DNA (cDNA) reverse transcription kit (Takara, Tokyo, Japan) was employed to synthesize cDNA from total RNA. SYBR Green Master Mix (Roche, Basel, Switzerland) was employed to perform RT-qPCR on the ABI 7500 cycler (Applied Biosystems, Foster City, CA, USA). Glyceraldehyde-3-phosphate dehydrogenase (GAPDH) was applied as a loading control for mRNA, with U6 for miRNA. N = 3. Analysis of the results was via 2^−ΔΔCt^. Primer sequences were manifested in Table 1.

**Table 1.** RT-qPCR primer sequence

	Primer sequence (5 ' – 3')
GAPDH	Forward: 5ʹ-CAGCCTCAAGATCATCAGCA-3’
	Reverse: 5ʹ-TGTGGTCATGAGTCCTTCCA-3’
U6	Forward: 5ʹ-CTCGCTTCGGCAGCACATATACT-3’
	Reverse: 5ʹ-ACGCTTCACGAATTTGCGTGTC-3’
MiR-129-5p	Forward: 5ʹ- GATCCGCAAGCCCAGACCGCAAAAAGTTTTTA-3’
	Reverse: 5ʹ-AGCTTAAAAACTTTTTGCGGTCTGGGCTTGCG −3’
DDX3X	Forward: 5ʹ- GAAAATGGAAGATATGGCCGTCG −3’
	Reverse: 5ʹ- TTCAGCACCACCATAAACCACG −3’
LncZFY-AS1	Forward: 5ʹ-TGTGAACCAGGTTTGCTGGA-3’
	Reverse: 5ʹ- CTCAACCATGCCGACGAGAA −3’

### 2.12 Western blot

Application of Radio-Immunoprecipitation assay buffer (Beyotime, Shanghai, China) was to extract total protein from cells or tissues. Separation of the same protein samples was via 10% sodium dodecyl sulfate polyacrylamide gel electrophoresis, and then electro-blot was onto Polyvinylidene fluoride membrane (Bio-Rad, Inc., Hercules, CA, USA). Then, after seal of the membrane with 5% skimmed milk, incubation was with Bax (1:1,000, ab32503), Bcl-2 (1:1000, ab32124), hypoxia-inducible factor 3 alpha (HIF3A) (1:1,000, ab10134), caspase-3 (1:1,000, ab32351) (Abcam, Cambridge, UK) and GAPDH (1:1000, 2118, Cell Signaling Technology), and secondary antibody (1:5,000, ab6728, Abcam). The immunoblotting was quantified via ImageLab software (Bio-Rad, Inc., Hercules, CA, USA). The protein concentration was normalized to GAPDH.

### 2.13 The luciferase activity assay

The LncZFY-AS1/DDX3X fragment consisting of miR-129-5p wild-type (WT) or mutant (MUT) binding site was cloned into pGL3 vector (Promega, Madison, WI, USA) to generate WT/mutant luciferase reporter vectors (WT-LncZFY-AS1/WT-DDX3X)/(MUT-LncZFY-AS1/MUT-DDX3X). Subsequently, transfection of the above vector and mimic-NC/miR-129-5p-mimic was into hPDLCs via Lipofectamine 3000 (Invitrogen, Carlsbad, CA, USA) obeying the protocol of the kit. Detection of the luciferase activity was via the dual luciferase reporter gene detection kit (Promega).

The article "Long non-coding RNA ZFY-AS1 represses periodontitis tissue inflammation and oxidative damage via modulating microRNA-129-5p/DEAD-Box helicase 3 X-linked axis" was retracted in 2026. Reasons: concerns about the data; concerns about the results or conclusions.

### 2.14 RNA immunoprecipitation (RIP) assay

Performance of RIP assay was as set forth [26]. RIP kit (Millipore, USA) was applied for RIP analysis. Lysis of hPDLCs was with RIP lysis buffer. Incubation of the lysate was with magnetic beads coupled with Ago2 or IgG antibody (Sigma, USA) in RIP buffer. Analysis of lncZFY-AS1, miR-129-5p and DDX3X was via RT-qPCR.

### 2.15 Data analysis

Processing of the statistical data was via SPSS 19.0 software (SPSS Inc., Chicago, IL, USA). One-way analysis of variance (ANOVA) or student’s t test was applied for comparison of differences of groups. Manifestation of the data was as mean ± standard deviation (SD). *P* < 0.05 emphasized obvious statistical meaning. Each experiment was carried out three biological replicates (N = 3).

## 3. Results

### 3.1 Knockdown lncZFY-AS1 refrains oxidative stress and inflammation in periodontitis mice

As clarified in Figure 1(a), lncZFY-AS1 was memorably elevated in periodontitis. Subsequently, LncZFY-AS1 in the periodontitis group was knocked down via injection of a short hairpin RNA lentiviral vector targeting lncZFY-AS1 (Figure 1(b)). It was clarified that *Pg* oral infection led to an elevation in the apoptosis rate of gingival tissue cells, which was then reduced via knocking down lncZFY-AS1 (Figure 1(c)). Subsequently, macrophage-specific marker F4/80 was checked to detect macrophage infiltration. It came out in Figure 1(d), *Pg* oral infection elevated the number of F4/80 positive cells in the gingival tissue, while knocking down lncZFY-AS1 decreased it. In the meantime, *Pg* oral infection facilitated inflammatory factors TNF-α, IL-1β and IL-6, while knocking down lncZFY-AS1 reduced them (Figure 1(e)). Subsequently, detection of NF-κB inflammation signal pathway was conducted. As manifested in Figure 1(f), *Pg* oral infection enhanced phosphorylated NF-κB and IκB in the gingival tissue, but repressive lncZFY-AS1 repressed them. Subsequently, examination of the effect of repressive lncZFY-AS1 was on the oxidative stress of the gingival tissue. As manifested in Figure 1(g), *Pg* oral infection strengthened peroxidation product MDA in the gingival tissue, but reduced antioxidant enzymes SOD and CAT, while knocking down lncZFY-AS1 was opposite. Meanwhile, *Pg* oral infection curbed antioxidant enzymes nuclear factor-E2-related factor 2 (Nrf2) and heme oxygenase 1 (HO-1), which was recovered via repressive lncZFY-AS1 (Figure 1(h)). These results affirmed that *Pg* oral infection accelerated the death of gingival tissue cells and resulted in severe oxidative damage and inflammation, while knocking down lncZFY-AS1 apparently mitigated the gingival tissue damage induced via *Pg* oral infection.

The article "Long non-coding RNA ZFY-AS1 represses periodontitis tissue inflammation and oxidative damage via modulating microRNA-129-5p/DEAD-Box helicase 3 X-linked axis" was retracted in 2026. Reasons: concerns about the data; concerns about the results or conclusions.

**Figure 1.** Knockdown lncZFY-AS1 represses oxidative stress and inflammation in mice with periodontitis a: RT-qPCR to detect lncZFY-AS1 in the gingival tissue of patients with periodontitis and the gingival tissue of mice; b: RT-qPCR to detect lncZFY-AS1 in the gingival tissue of mice transfected with sh-lncZFY-AS1 lentiviral vector; c: TUENL staining examination of mouse gingival cell apoptosis after knocking down lncZFY-AS1; d: Immunohistochemical detection of macrophage specific marker F4/80 after knocking down lncZFY-AS1; e: The effect of repressive lncZFY-AS1 on the inflammatory factors TNF-α, IL-1β and IL-6 in the gingival tissue of mice; F: Western blot detection of the effect of knocking down lncZFY-AS1 on phosphorylated NF-κB and IκB; g: The effect of depressive lncZFY-AS1 on the oxidative stress factors MDA, SOD and CAT in mouse gingival tissue; h: Western blot to detect the effect of repressive lncZFY-AS1 on HO-1 and Nrf2 proteins; The data were manifested as mean ± SD (n = 6); * *P* < 0.05.

### 3.2 Enhancive lncZFY-AS1 motivates cell inflammation and oxidative stress in hPDLCs

For exploring the latent molecular mechanism of lncZFY-AS1 in periodontitis, *in vitro* experiments were conducted then. Establishment of the periodontitis cell model was via LPS treatment of hPDLCs. As manifested in Figure 2(a), LPS treatment obviously elevated lncZFY-AS1 in hPDLCs, and transfection with pcDNA 3.1-lncZFY-AS1 further enhanced it. Some experiments clarified that LPS treatment reduced the advancement of hPDLCs, while elevated lncZFY-AS1 further enhanced the impacts (Figure 2(b,c)). Subsequently, check of inflammatory factors was manifested. As clarified in Figure 2(d,e), LPS treatment elevated TNF-α, IL-1β, IL-6, and phosphorylated NF-κB and IκB in hPDLCs, which was further strengthened via enhancive lncZFY-AS1. Next, it was checked the oxidative stress. As manifested in Figure 2(f,g), LPS treatment enhanced MDA in hPDLCs, but reduced SOD, CAT, Nrf2 and HO-1, while elevated lncZFY-AS1 aggravated this effect. These results emphasized that enhancive lncZFY-AS1 could aggravate the apoptosis, inflammation and oxidative damage of hPDLCs induced via LPS.

**Figure 2.** Enhancive lncZFY-AS1 facilitates cell inflammation and oxidative stress in hPDLCs a: RT-qPCR to detect lncZFY-AS1 after elevated lncZFY-AS1; b: MTT to detect the effect of elevated lncZFY-AS1 on cell viability; c: Flow cytometry detection of the effect of elevated lncZFY-AS1 on cell apoptosis; d: The effect of elevated lncZFY-AS1 on the inflammatory factors TNF-α, IL-1β and IL-6; e: Western blot detection of the effect of elevated lncZFY-AS1 on phosphorylation of NF-κB and IκB; f: The effect of elevated lncZFY-AS1 on MDA, SOD and CAT; g: Western blot detection of the effect of elevated lncZFY-AS1 on HO-1 and Nrf2 proteins; In hPDLCs; The data were manifested as mean ± SD (n = 3); * *P* < 0.05.

The article "Long non-coding RNA ZFY-AS1 represses periodontitis tissue inflammation and oxidative damage via modulating microRNA-129-5p/DEAD-Box helicase 3 X-linked axis" was retracted in 2026. Reasons: concerns about the data; concerns about the results or conclusions.

### 3.3 Elevated miR-129-5p represses cell inflammation and oxidative stress in hPDLCs

RT-qPCR was applied to check the expression of miR-129-5p in periodontitis. As shown in Figure 3(a). The expression of miR-129-5p in periodontitis patients, mice and cell models was all reduced vs. normal controls. Subsequently, miR-129-5p expression was up-regulated or down-regulated by transfection of miR-129-5p-mimic/inhibitor into hPDLCs (Figure 3(b)). Functional assay studies manifested overexpression of miR-129-5p elevated the cell viability of hPDLCs (Figure 3(c)), decreased the apoptosis rate of hPDLCs cells (Figure 3(d)), refrained the release of TNF-α, IL-1β and IL-6 (Figure 3(e)) and the protein expression of phosphorylated NF-κB and IκB (Figure 3(f)), reduced the MDA level of hPDLCs cells, elevated SOD and CAT levels (Figure 3(g)), and promoted the protein expression of Nrf2 and HO-1 (Figure 3(h)), while the knockdown of miR-129-5p had completely opposite effects. These results suggested miR-129-5p repressed inflammation and oxidative stress in hPDLCs.

**Figure 3.** Elevated miR-129-5p refrains hPDLCs inflammation and oxidative stress a: RT-qPCR to detect the expression of miR-129-5p in periodontitis patients, mice and cell models; b: RT-qPCR to detect the expression of miR-129-5p in hPDLCs after transfection with miR-129-5p-mimic/inhibitor; c: Effects of transfection with miR-129-5p-mimic/inhibitor on hPDLCs viability detected by MTT; d: Flow cytometry to detect the effect of transfection with miR-129-5p-mimic/inhibitor on apoptosis of hPDLCs cells. e: Effects of transfection with miR-129-5p-mimic/inhibitor on hPDLCs inflammatory factors TNF-α,IL-1β and IL-6; f: Western blot analysis of the effects of transfection with miR-129-5p-mimic/inhibitor on the expression of phosphorylated NF-κB and IκB protein in hPDLCs; g: Effects of transfection with miR-129-5p-mimic/inhibitor on MDA, SOD and CAT in hPDLCs; h: Western blot to detect the effects of transfection with miR-129-5p-mimic/inhibitor on the protein expression of HO-1 and Nrf2 in hPDLCs. The data were represented by mean ± SD (n = 3). * P < 0.05.

### 3.4 LncRNA ZFY-AS1 competitively combines with miR-129-5p

LncRNA usually competitively adsorbs miRNAs to play a modulatory role in cell post-transcriptional expression. Next, it was checked whether lncZFY-AS1 targeted miR-129-5p. As manifested in Figure 4(a), knockdown lncZFY-AS1 elevated miR-129-5p in mouse gingival tissues, while enhancive one refrained it in hPDLCs. This indicated that miR-129-5p was modulated via lncZFY-AS1. Next, it was checked the targeting of lncZFY-AS1 with miR-129-5p. Through the bioinformatics website https://cm.jefferson.edu/, was predicted that lncZFY-AS1 and miR-129-5p had potential binding sites (Figure 4(b)). Subsequently, an experiment was performed to further verify the targeting of them. As manifested in Figure 4(c), the luciferase activity was obviously reduced after the co-transfection of WT LncZFY-AS1 and miR-129-5p-mimic, but the co-transfection of mutant lncZFY-AS1 and miR-129-5p-mimic did not affect it. Additionally, it was detected that lncZFY-AS1 and miR-129-5p were enriched in the precipitate (Figure 4(d)). The results confirmed that lncZFY-AS1 competitively absorbed miR-129-5p.

The article "Long non-coding RNA ZFY-AS1 represses periodontitis tissue inflammation and oxidative damage via modulating microRNA-129-5p/DEAD-Box helicase 3 X-linked axis" was retracted in 2026. Reasons: concerns about the data; concerns about the results or conclusions.

**Figure 4.** LncZFY-AS1 competitively combines with miR-129-5p a: RT-qPCR to detect miR-129-5p in mouse gingival tissues or hPDLCs after repressive or elevated lncZFY-AS1; b: The binding sites of lncZFY-AS1 and miR-129-5p predicted by bioinformatics websites; c: The luciferase activity assay to detect the targeting of lncZFY-AS1 and miR-129-5p; d: RIP assay to detect the binding of lncZFY-AS1 and miR-129-5p; The data were manifested as mean ± SD (n = 3); * *P* < 0.05.

### 3.5 LncZFY-AS1 influences inflammation and oxidative stress in hPDLCs via modulating miR-129-5p

Next, it was explored whether miR-129-5p was linked with the biological role of lncZFY-AS1 in hPDLCs. The si-lncZFY-AS1 and miR-129-5p-inhibitor were co-transfected into hPDLCs. It was indicated that transfection of si-lncZFY-AS1 elevated miR-129-5p in hPDLCs, while co-transfection of miR-129-5p-inhibitor prevented the up-regulation of miR-129-5p (Figure 5(a)). The experiments clarified that transfection of si-lncZFY-AS1 strengthened hPDLCs advancement, and repressed inflammatory factors TNF-α, IL-1β and IL-6 and phosphorylated NF-κB and IκB, MDA, and elevated SOD, CAT, HO-1 and Nrf2, while co-transfection of miR-129-5p-inhibitor reversed this phenomenon (Figure 5(b-g)). The results clarified that lncZFY-AS1 accelerated hPDLCs inflammation and oxidative stress via modulating miR-129-5p.

**Figure 5.** LncZFY-AS1 affects hPDLCs inflammation and oxidative stress via modulating miR-129-5p a: RT-qPCR to detect miR-129-5p in hPDLCs after co-transfection; b: MTT to detect the effect of co-transfection of si-lncZFY-AS1 and miR-129-5p-inhibitor on hPDLCs viability; c: Flow cytometry to detect the effect of co-transfection of si-lncZFY-AS1 and miR-129-5p-inhibitor on hPDLCs apoptosis; d: The effect of co-transfection of si-lncZFY-AS1 and miR-129-5p-inhibitor on the inflammatory factors TNF-α, IL-1β and IL-6 in hPDLCs; e: Western blot detection of the effect of co-transfection of si-lncZFY-AS1 and miR-129-5p-inhibitor on phosphorylated NF-κB and IκB in hPDLCs; f: The effect of co-transfection of si-lncZFY-AS1 and miR-129-5p-inhibitor on MDA, SOD and CAT in hPDLCs; g: Western blot to detect the effect of co-transfection of si-lncZFY-AS1 and miR-129-5p-inhibitor on HO-1 and Nrf2 proteins in hPDLCs; The data were manifested as mean ± SD (n = 3); * *P* < 0.05.

The article "Long non-coding RNA ZFY-AS1 represses periodontitis tissue inflammation and oxidative damage via modulating microRNA-129-5p/DEAD-Box helicase 3 X-linked axis" was retracted in 2026. Reasons: concerns about the data; concerns about the results or conclusions.

### 3.6 DDX3X is the target gene of miR-129-5p

Next, it was explored the target genes of miR-129-5p. DDX3X is the upstream modulator of inflammasome NLRP3 [27]. In this study, it was discovered that DDX3X was up-regulated in periodontitis (Figure 6(a)). Additionally, repressive or enhancive DDX3X was found in hPDLCs with up-regulated or down-regulated miR-129-5p (Figure 6(b)). This indicated that DDX3X was controlled via miR-129-5p. Then it was explored the targeting of DDX3X with miR-129-5p. Via the bioinformatics website http://starbase.sysu.edu.cn/, was forecast that DDX3X and miR-129-5p had latent binding sites (Figure 6c). Subsequently, some experiments were conducted to further verify the targeting of them. The results affirmed that co-transfection of WT DDX3X and miR-129-5p-mimic would reduce the luciferase activity, while that of mutant DDX3X and miR-129-5p-mimic had no impacts on the luciferase activity (Figure 6(d)). In the meantime, an experiment affirmed that DDX3X and miR-129-5p were clearly enriched in the precipitate (Figure 6(e)). These results suggested that DDX3X was the target gene of miR-129-5p.

**Figure 6.** DDX3X is the target gene of miR-129-5p a: Western blot to detect DDX3X in periodontitis patients, mice and cell models; b: Western blot detection of DDX3X in hPDLCs after up-regulation or down-regulation of miR-129-5p; c: Binding sites of DDX3X and miR-129-5p predicted by bioinformatics sites; d: The luciferase activity assay to detect the targeting of DDX3X and miR-129-5p; e: RIP assay to detect the binding of DDX3X and miR-129-5p; The data were manifested as mean ± SD (n = 3); * *P* < 0.05.

### 3.7 LncZFY-AS1 modulates hPDLCs inflammation and oxidative stress via modulating miR-129-5p/DDX3X pathway

Next, through functional rescue experiments, it was explored whether the miR-129-5p/DDX3X axis was involved in the process of lncZFY-AS1 modulating hPDLCs inflammation and oxidative stress. The si-lncZFY-AS1 and pcDNA 3.1-DDX3X were co-transfected into hPDLCs and DDX3X was checked. As clarified in Figure 7(a), DDX3X with transfected si-lncZFY-AS1 was reversed by co-transfection of pcDNA 3.1-DDX3X. Other experiments manifested that transfection of si-lncZFY-AS1 accelerated cell viability, while co-transfection of pcDNA 3.1-DDX3X prevented this phenomenon (Figure 7(b)). Moreover, transfection of si-LncZFY-AS1 reduced the rate of apoptosis, which was recovered via co-transfection of pcDNA 3.1-DDX3X (Figure 7(c)). Subsequently, the effect of co-transfection on cell inflammation and oxidative stress was examined. As manifested in Figure 7(d-g), transfection of si-lncZFY-AS1 clearly reduced inflammatory factors, MDA and phosphorylated NF-κB and IκB, but elevated SOD, CAT, HO-1 and Nrf2, but co-transfection with pcDNA 3.1-DDX3X turned around this phenomenon. The results clarified that lncZFY-AS1 modulated hPDLCs inflammation and oxidative stress via modulating miR-129-5p/DDX3X pathway.

The article "Long non-coding RNA ZFY-AS1 represses periodontitis tissue inflammation and oxidative damage via modulating microRNA-129-5p/DEAD-Box helicase 3 X-linked axis" was retracted in 2026. Reasons: concerns about the data; concerns about the results or conclusions.

**Figure 7.** LncZFY-AS1 controls hPDLCs inflammation and oxidative stress through miR-129-5p/DDX3X pathway a: Western blot to detect DDX3X in hPDLCs after co-transfection of si-lncZFY-AS1 and pcDNA 3.1-DDX3X; b: MTT assay to detect the effect of co-transfection of si-lncZFY-AS1 and pcDNA 3.1-DDX3X on hPDLCs viability; c: Flow cytometry to detect the effect of co-transfection of si-lncZFY-AS1 and pcDNA 3.1-DDX3X on apoptosis of hPDLCs; d: Effects of co-transfection of si-lncZFY-AS1 and pcDNA 3.1-DDX3X on inflammatory cytokines TNF-α, IL-1β and IL-6 in hPDLCs; e: Western blot analysis of the effects of co-transfection of si-lncZFY-AS1 and pcDNA 3.1-DDX3X on phosphorylated NF-κB and IκB proteins in hPDLCs; f: Effects of co-transfection of si-lncZFY-AS1 and pcDNA 3.1-DDX3X on MDA, SOD and CAT in hPDLCs; g: Western blot analysis of the effects of co-transfection of si-lncZFY-AS1 and pcDNA 3.1-DDX3X on HO-1 and Nrf2 proteins in hPDLCs; The data were manifested as mean ± SD (n = 3); * *P* < 0.05.

## 4. Discussion

Long-term chronic periodontitis is available to cause serious inconvenience to patients’ lives, and current treatments for periodontitis have limited effects on improving patients’ lives [28]. Therefore, it is necessary to further understand the molecular mechanism of periodontitis. In this study, it was discovered that a non-coding RNA called lncZFY-AS1 is crucial in the pathogenesis of periodontitis. Knockdown lncZFY-AS1 effectively mitigated periodontitis tissue inflammation and oxidative stress, and accelerated hPDLCs viability and reduced apoptosis. In terms of mechanism, repressive lncZFY-AS1 reduced NF-κB inflammation signaling pathway protein, and accelerated antioxidant signaling pathway Nrf2/HO-1 protein to relieve periodontitis via competitively combining with miR-129-5p and depressing DDX3X.

The article "Long non-coding RNA ZFY-AS1 represses periodontitis tissue inflammation and oxidative damage via modulating microRNA-129-5p/DEAD-Box helicase 3 X-linked axis" was retracted in 2026. Reasons: concerns about the data; concerns about the results or conclusions.

In the middle and late stages of chronic tissue inflammation (such as periodontitis), the inflammatory stimulus will be sensed by macrophages, inducing infiltration into the tissue and stimulating downstream cascade signal responses [29,30]. Previous studies have clarified that lncRNA functions in modulating the inflammatory response of macrophages. These lncRNAs consist of lncMEG3 [31], lncH19 [32] and lncAFAP1-AS1 [33], etc. In this study, it was first examined the role of lncRNA in controlling the infiltration of periodontitis macrophages. Depressive lncZFY-AS1 reduced macrophage-specific marker F4/80 in mouse gingival tissue. Additionally, it was discovered that knocking down lncZFY-AS1 reduced inflammatory factors TNF-α, IL-1β, and IL-6 in the periodontitis model. It is worth noting that these inflammatory factors are mainly released by macrophages under inflammatory stimulation [34]. Therefore, it was speculated that preventing macrophage infiltration is a momentous measure for lncZFY-AS1 to repress periodontitis inflammation. A great many studies have proved that lncRNA can modulate the phenotype of macrophages. For example, lncPVTA refrains the polarization of macrophages M1 to alleviate sepsis-induced myocardial inflammation [35]. LncH19 accelerates the polarization of macrophage M1 to aggravate arthritis [36]. It was speculated that lncZFY-AS1 motivating periodontitis tissue inflammation might be linked with the modulation of macrophage polarization. But this needs to be further explored in a follow-up study.

Subsequently, it was further confirmed that miR-129-5p/DDX3X was a key pathway for lncZFY-AS1 to regulate hPDLCs cell damage through dual-luciferase reporting assay, RIP assay and functional rescue assay. Previous studies have manifested miR-129-5p performs cleavage or direct translation repression by binding to the 3ʹuntranslated region of target gene mRNAs such as HMGB1 [37] and Keap-1 [38], thus playing a role in tissue inflammation and oxidative damage. In this study, overexpression of miR-129-5p reduced LPS-induced inflammation, oxidative damage and apoptosis of hPDLCs. These data further support miR-129-5p is a momentous factor in body immune regulation. In addition, in this study, it was found that DDX3X was the downstream target gene of miR-129-5p. Repressive lncZFY-AS1’s depression on inflammation, oxidative damage and apoptosis of hPDLCs was reversed via elevated DDX3X, which suggested that DDX3X was a key protein modulated by lncZFY-AS1 in periodontitis.

The NF-κB signaling pathway is vital in the inflammation and immune response of periodontal tissues [39]. IκB is a repressive protein of NF-κB and restrains its activity via binding to NF-κB [40,41]. Former studies have affirmed that lncRNA (such as lncNron7, lncFGD5-AS123) accelerates or depresses inflammation via modulating the activity of NF-κB in gum tissue. In this study, it was discovered that knocking down LncZFY-AS1 repressed the phosphorylation of NF-κB and motivated the phosphorylation of IκB. This clarified that lncZFY-AS accelerated periodontitis inflammation via activating the NF-κB pathway. For further understanding its molecular mechanism, a functional rescue experiment was conducted. The results manifested that the effect of repressive lncZFY-AS was reversed by restrained miR-129-5p or elevated DDX3X. A former study clarifies that DDX3X mediates NLRP3 inflammasome activation [27]. NLRP3 inflammasome is strictly controlled by NF-κB signaling [42]. This manifests that lncZFY-AS may activate NF-κB and induce the activation of NLRP3 inflammasomes via controlling the miR-129-5p/DDX3X axis. It is necessary to further explore it in subsequent research, which is conducive to a more comprehensive understanding of the pathogenesis of periodontitis.

The article "Long non-coding RNA ZFY-AS1 represses periodontitis tissue inflammation and oxidative damage via modulating microRNA-129-5p/DEAD-Box helicase 3 X-linked axis" was retracted in 2026. Reasons: concerns about the data; concerns about the results or conclusions.

The Nrf2/HO-1 signaling pathway is a classic antioxidant pathway. Nrf2 scavenges reactive oxygen species via formation of a heterodimer with the Maf protein through the Neh1 domain and combination with the phase II detoxification enzyme HO-1 [43]. This is conducive to modulating the balance of cellular oxidative stress, apoptosis and inflammation, and other cellular activities [44,45]. A former study clarifies that lncJHDM1D-AS1 protects H_2_O_2_ to induce parodontium stem cell apoptosis and reduce ROS [46]. Here, it was demonstrated for the first time that lncZFY-AS reduces antioxidant enzymes and accelerates the oxidative damage of PDLCs via repressing the Nrf2/HO-1 pathway. Additionally, the motivating effect of lncZFY-AS on oxidative stress will further enhance inflammatory damage.

Although the results of this study suggest lncZFY-AS1/miR-129-5p/DDX3X may serve as a potential molecular target for the treatment of periodontitis, it is necessary to further understand whether lncZFY-AS1 is supposed to serve as a potential biomarker of periodontitis, which will contribute to the early diagnosis of periodontitis. Therefore, serum expression of lncZFY-AS1 and ROC clinical data need to be monitored in subsequent studies. In addition, whether lncZFY-AS1/miR-129-5p/DDX3X can be applied as a therapeutic target for patients with periodontitis requires to be verified in clinical studies.

## 5. Conclusion

All in all, the results of this study clarify that lncZFY-AS modulates the Nrf2/HO-1 and NF-κB signaling pathways in periodontitis via competitively adsorbing miR-129-5p to mediate DDX3X, which helps to facilitate the deterioration of periodontitis. LncZFY-AS/miR-129-5p/DDX3X axis is supposed to be applied as an information target for the treatment of periodontitis later.
